# *TaWRKY40* transcription factor positively regulate the expression of *TaGAPC1* to enhance drought tolerance

**DOI:** 10.1186/s12864-019-6178-z

**Published:** 2019-10-30

**Authors:** Lin Zhang, Zhiyong Xu, Haikun Ji, Ye Zhou, Shushen Yang

**Affiliations:** College of Life Sciences, Northwest A&F University, Yangling, 712100 Shaanxi China

**Keywords:** *Triticum aestivum*, *TaGAPC1*, *TaWRKY40*, Drought

## Abstract

**Backgrounds:**

Drought stress is one of the major factors that affects wheat yield. Glyceraldehyde-3-Phosphate dehydrogenase (GAPDH) is a multifunctional enzyme that plays the important role in abiotic stress and plant development. However, in wheat, limited information about drought-responsive GAPC genes has been reported, and the mechanism underlying the regulation of the GAPC protein is unknown.

**Results:**

In this study, we evaluated the potential role of *GAPC1* in drought stress in wheat and Arabidopsis. We found that the overexpression of *TaGAPC1* could enhance the tolerance to drought stress in transgenic Arabidopsis. Yeast one-hybrid library screening and EMSA showed that TaWRKY40 acts as a direct regulator of the *TaGAPC1* gene. A dual luciferase reporter assay indicated that TaWRKY40 improved the *TaGAPC1* promoter activity. The results of qRT-PCR in wheat protoplast cells with instantaneous overexpression of *TaWRKY40* indicated that the expression level of *TaGAPC1* induced by abiotic stress was upregulated by TaWRKY40. Moreover, *TaGAPC1* promoted H_2_O_2_ detoxification in response to drought.

**Conclusion:**

These results demonstrate that the inducible transcription factor TaWRKY40 could activate the transcription of the *TaGAPC1* gene, thereby increasing the tolerance of plants to drought stress.

## Background

Plant environmental stresses include drought, salt, extreme climate and oxidative stress, which seriously threaten food security and agricultural production. Due to global climate change, the environmental stress on plants will be increased over the next few years [1]. However, most crops, such as wheat, rice and tomato, are sensitive to drought stress. Therefore, it is necessary to study the stress resistance of crop plants and to adapt plants to a stressful growth environment [2].

For a long time, GAPDH has been used as a housekeeping gene in gene expression analysis [3]. The GAPDH gene family is conserved across different living organisms, and the family of genes plays a vital role in carbon metabolism in the cell [4]. In plant cells, GAPDH participates in glycolysis and the Calvin cycle in different forms and in different locations [5]. GAPDHs are classified into three groups according to their different subcellular locations in plant cells, namely, GAPA/B, GAPC and GAPCp, and the functions of these proteins in some plant growth mechanisms have been revealed [6–8]. Some studies have shown that GAPDH acts as a non-glycolytic functional protein. GAPDH appears to have suitable properties to behave as an oxidative stress sensor in plant cells, and this function has no relationship with its classical glycolytic role. In Arabidopsis, oxidatively modified cytoplasmic GAPDH has been successfully used as a tool to investigate the role of reduced glutathione, thioredoxins and glutaredoxins in the control of different types of redox post-translational modifications [9]. The aggregation of GAPDH in the cytoplasm, which may be induced by oxidative stress, was associated with cell death [10]. Similarly, in the pea plant, GAPDH was also associated with programmed cell death and seed ageing [11]. In addition, several studies have shown that GAPC is also involved in signal transduction when plants are suffering from abiotic stress. In Arabidopsis, cytosolic GAPC participates in the signal cascade induced by ROS by interacting with H_2_O_2_ [12]. In Arabidopsis GAPC mutants, an imbalance of amino acids and carbohydrates leads to impaired ABA signaling, which subsequently affects ABA signaling pathways and the primary metabolism of plants [13]. GAPC1 relocated to the nucleus as result of oxidative stress-induced signal transduction where it performed its secondary functions when plants were suffering from cadmium treatments [14]. Furthermore, different types of redox modifications of GAPC in Arabidopsis could help control the flexibility of GAPC function, allowing it to participate in diverse cellular processes and pathways [15]. In Arabidopsis, GAPC1 translocated into the nucleus in a process mediated by SINAL7 which had a positive effect on vegetative growth, thereby reducing the flux of glycolytic pathways in the cytoplasm, and performing non-glycolytic functions in the nucleus [16, 17]. A deficiency in GAPC activity could improve the seed numbers and embryo development by modifying carbon flux and mitochondrial dysfunction, suggesting that *GAPC1* is vital to normal fertility in Arabidopsis plants [18].

In wheat, four types of GAPDHs (gapA/B, gapC, gapCp and gapN) including 22 *GAPDH* genes were identified, and qRT-PCR results indicated that *GAPDHs* showed different expression levels under the conditions of several abiotic stresses [19]. However, the potential roles of wheat *GAPC* genes in response to abiotic stress including drought have not been evaluated. Here, we showed that *TaGAPC1* positively regulated drought stress tolerance in Arabidopsis. A WRKY transcription factor TaWRKY40 in wheat was screened by a yeast one-hybrid system. An electrophoretic mobility shift assay (EMSA) confirmed that TaWRKY40 could directly bind to the *TaGAPC1* promoter. The expression level of *TaGAPC1* was significantly higher under drought stress in wheat protoplast cells with instantaneous overexpression of *TaWRKY40* than in wild type wheat protoplast cells. These results demonstrated that TaWRKY40 may positively regulate the *TaGAPC1* expression. The high expression level exhibited by TaWRKY40 may be an important clue to investigate the secondary functions of TaGAPC1.

## Results

### Expression profile of *TaGAPC1* in response to abiotic stress and subcellular localization of TaGAPC1

To clarify potential functions, the responses of *TaGAPC1* to various abiotic stress conditions were analyzed by qRT-PCR (Fig. 1a). The results showed that *TaGAPC1* expression increased to a maximum level of approximately five-fold after 6 h of PEG treatment. *TaGAPC1* gene responded to ABA, with the peak level (more than 9-fold) occurring after 4 h of treatment. *TaGAPC1* showed response to H_2_O_2_ stress, peaking at more than 7-fold. These results indicated that the transcriptional level of *TaGAPC1* was significantly affected by abiotic stress. In addition to seeds, *TaGAPC1* was highly expressed in almost all tissues including roots, stems and leaves (Fig. 1b).

**Fig. 1:** *TaGAPC1* expression in response to abiotic stresses in wheat and protein localization. **a** Time-course expression of *TaGAPC1* in in wheat. **b** Tissue-specific expression pattern of *TaGAPC1* in wheat. 1 and 2 Two-leaf stage (leaf and root), 3 and 4 Tillering stage (leaf and root), 5 and 6 Jointing stage (leaf and root), 7 and 8 Heading stage (leaf and root), 9 Seed. Error bars indicate ±SD (*n* = 3, from three technical replicates). Significant differences were assessed with one-sided paired t-tests (*, *P* < 0.05; **, *P* < 0.01). Three biological experiments were performed, which produced similar results. **c** TaGAPC1 is localized in the nucleus and cytoplasm of wheat protoplast cells, TaWRKY40 is localized in the nucleus of wheat protoplast cells. Bars, 100 μm

To further investigate the biological activity of TaGAPC1, fused *TaGAPC1*-GFP was transiently expressed in wheat protoplasts. In Fig. 1c, the wheat protoplast expressing 35S::*TaGAPC1*-GFP showed clear green fluorescence in the cytoplasm and nucleus. These results indicated that TaGAPC1 was located in both the cytoplasm and nucleus. The subcellular localization of TaGAPC1 was also consistent with previous reports that MeGAPCs [20], NbGAPCs [21], and AtGAPCs [22] have some nuclear localization.

### TaGAPC1 can enhance drought tolerance and stimulate H_2_O_2_ scavenging in transgenic Arabidopsis plants

To determine whether *TaGAPC1* gene is important for drought stress tolerance, we evaluated drought stress response in transgenic Arabidopsis plants overexpressing *TaGAPC1* gene (1014 bp) under the control of the strong 35S promoter. Arabidopsis plants overexpressing TaGAPC1 gene showed TaGAPC1 expression using pr1 and pr2 primer pair, and TaGAPC1-GFP fusion genes using the pr1 and pr3 primer pair, but no expression was observed in wild type (Additional file 1: Figure S1B and S1C) Transgenic lines expressing *TaGAPC1* showed a higher survival rate than Col-0 (wild type) after 25 days of withholding water. The contents of RWC and chlorophyll in the OE1–3 and OE1–10 lines were also higher than Col-0 after 15 days of drought stress (Fig. 2). Arabidopsis plants deficient in GAPCs were less sensitive to ABA-promoted stomatal closure than the Col-0 plants under drought stress [16]. Thus, we speculate that stomatal closure may be related to the increased drought tolerance observed in Arabidopsis plants overexpressing *TaGAPC1*. Expanded leaves from Arabidopsis plants after 15 days of drought stress were measured to determine the guard cell stomatal aperture. The guard cells of OE1–3 and OE1–10 were dramatically changed and the stomatal apertures of OE1–3 and OE1–10 were smaller than those of Col-0 plants (Fig. 3). These results indicated that *TaGAPC1* actively respond to plant drought stress.

**Fig. 2:** *TaGAPC1* responding to drought stress treatment in Arabidopsis. **a** Tolerance responses of the *TaGAPC1*–overexpressing (OE1–3 and OE1–10) lines to drought stress. Drought 15 d, withholding water for 15 d; Drought 25 d, with holding water for 25 d; R7 d, resumption of water for 7 d after withholding water for 25 d. **b** Survival rates of *TaGAPC1*–overexpressing (OE1–3 and OE1–10) transgenic lines, Col-0 and VC plants on day 7 after resuming water following the withholding of water for 25 d. At least 100 plants were counted and averaged for each line. **c** The chlorophyll content of Col-0 and *TaGAPC1*–overexpressing (OE1–3 and OE1–10) lines after withholding water for 15 d. **d** The MDA content of Col-0 and *TaGAPC1*–overexpressing (OE1–3 and OE1–10) lines after withholding water for 15 d. (E) RWC of Col-0 and *TaGAPC1*–overexpressing (OE1–3 and OE1–10) lines after withholding water for 15 d. Error bars indicate ±SD (*n* = 3, from three technical replicates). Significant differences were assessed with one-sided paired t-tests (*, *P* < 0.05; **, *P* < 0.01). Three biological experiments were performed, which produced similar results

**Fig. 3:** Analyze of stomatal aperture size. **a** Images of stomatal apertures from epidermal peels of Col-0 and *TaGAPC1*–overexpressing (OE1–3 and OE1–10) lines after withholding water for 15 d. Scale bars: 10um. **b** The stomatal aperture size was determined by measuring the width to length of stomates in epidermal peels from Col-0 and *TaGAPC1*–overexpressing (OE1–3 and OE1–10) lines after withholding water for 15 d. Error bars indicate ±SD (*n* = 50). Significant differences were assessed with one-sided paired t-tests (*, *P* < 0.05; **, *P* < 0.01). Three biological experiments were performed, which produced similar results

The overproduction of reactive oxygen species (ROS) is toxic to cellular processes and can disrupt the electron transport chain [23]. Thus, we detected ROS accumulation and physiological differences. NBT was used to test the level of O^2−^ in leaves after withholding water for 15 days. The leaves of OE1–3 and OE1–10 all had the weaker staining than those of Col-0 Arabidopsis (Fig. 4). Consistently, the H_2_O_2_ content of OE1–3 and OE1–10 were also lower than that of Col-0 after withholding water for 15 days. In plants, POD can scavenge H_2_O_2_ by hydroxylation. After withholding water for 15 days, the activity of POD was higher in *TaGAPC1-*overexpressing plants than in Col-0 plants. In addition, the activity of SOD, another antioxidant enzyme that catalyses the dismutation of the superoxide (O^2−^) radical into H_2_O_2_, also showed a similar pattern in transgenic plants after withholding water for 15 days (Fig. 4). These results indicated that *TaGAPC1* promoted ROS scavenging by modulating the activity of antioxidant enzymes, such as POD and SOD.

**Fig. 4:** *TaGAPC1* promote hydrogen peroxide (H_2_O_2_) scavenging in response to drought stress. **a** O^2−^ accumulation in Col-0 and *TaGAPC1*–overexpressing (OE1–3 and OE1–10) lines after withholding water for 15 d. O^2−^ was indicated by NBT staining. **b**–**d** H_2_O_2_ content, superoxide dismutase (SOD) and peroxidase (POD) activity in Col-0 and *TaGAPC1*–overexpressing (OE1–3 and OE1–10) lines after withholding water for 15 d. Error bars indicate ±SD (*n* = 3, from three technical replicates). Significant differences were assessed with one-sided paired t-tests (*, *P* < 0.05; **, *P* < 0.01). Three biological experiments were performed, which produced similar results

### TaGAPC1 promoter activity analysis

To further understand the regulation of *TaGAPC1* under abiotic stress, a 1500 bp promoter was cloned and analyzed by PLANTCARE and NEWPLACE. Bioinformatics analysis indicated that there were multiple cis-acting elements related to stress tolerance, such as MYB, W-BOX and other components (Fig. 5a). The promoter was fused to the PC0390 vector to drive GUS enzyme activity. As shown in Fig. 5b, the GUS staining results indicated that the promoter had activity in tobacco. The luciferase assay in the instantaneous transient tobacco line showed that the activity of the *TaGAPC1* promoter was significantly enhanced under abiotic stress. These results were consistent with the above results (Fig. 1). These observations suggested that *TaGAPC1* may be involved in the abiotic stress signal transduction of plants.

**Fig. 5:** Activity of *TaGAPC1* promoter after PEG8000, ABA and H_2_O_2_ abiotic stresses. **a** cis-elments of *TaGAPC1* promoter. **b** Histochemical staining of *TaGAPC1* promoter in transiently transformed tobacco leaves. P: positive control (CaMV 35S promoter); WT: wild type. **c** Analysis of RLUC activity for *TaGAPC1* promoter in transiently transformed tobacco leaves in response to stress. Error bars indicate ±SD (*n* = 3, from three technical replicates). Significant differences were assessed with one-sided paired t-tests (*, *P* < 0.05; **, *P* < 0.01). Three biological experiments were performed, which produced similar results

### TaWRKY40 can interact with the TaGAPC1 promoter in vivo and in vitro

To gain more insight into the *TaGAPC1* - mediated drought response, we identified the proteins that interact with the *TaGAPC1* promoter through a genome-wide yeast one-hybrid screen with a cDNA library. Through selection on SD/-Leu + AbA medium and DNA sequencing, 33 proteins were identified as candidate proteins that interact with *TaGAPC1* promoter (Additional file 4: Table S2). Among the 33 potential candidate proteins, TaWRKY40 was of the great interest. Recent studies have shown that WRKYs could take part in several signal transduction pathways involved in plant abiotic stress. The W box (T/CTGACC/T) is the targeted cis-element of the WRKY transcription factor [24]. There are six putative W box elements in the *TaGAPC1* promoter. To examine which W box is the targeted cis-element of TaWRKY40, six *TaGAPC1* promoter fragments containing the W box (Additional file 3: Table S1), as shown in Fig. 6a, were cloned into the bait vector of pAbAi, and the coding sequence of *TaWRKY40* was cloned into the prey vector of pGADT7. After co-transformation into yeast for the Y1H assay, we found that TaWRKY40 activated the *TaGAPC1* promoter constructs (− 708--836, − 290—426, − 160--289) in yeast, as evidenced by the growth of the transformant clone in on selective SD/-Leu + AbA medium (Fig. 6).

**Fig. 6:** *TaWRKY40* directly binds to the promoter region of *TaGAPC1*. **a** Schematic diagram of the probe used for Electrophoretic mobility shift assays (EMSA). Probe1, 2, 3, 4, 5 and 6 contain W-box, whereas in the probe1–1, 2–1, 3–1, 4–1, 5–1 and 6–1, the W-box core sequence was mutated. The mutated bases are indicated in red. **b** Schematic diagrams of the effector and reporter used for transient transactivation assays in tobacco. **c** Yeast one-hybrid confirm the interaction. **d** Transactivation activity reflected by RLUC activity of RLUC/FLUC ratio. Pro35S: GUS was used as an internal control. Quantification was performed by normalizing Firefly luciferase activity to that of Renilla luciferase. **e** *TaWRKY40* binding specific W-box motifs by EMSA. Error bars indicate ±SD (*n* = 3, from three technical replicates). Significant differences were assessed with one-sided paired t-tests (*, *P* < 0.05; **, *P* < 0.01). Three biological experiments were performed, which produced similar results

To further determine whether the TaWRKY40 protein directly bound to the *TaGAPC1* promoter in vitro, we performed electrophoretic mobility shift assays (EMSA) using a promoter fragment of approximately 40 bp as a probe. The results showed that TaWRKY40 could specifically bind to these W box in *TaGAPC1* promoter fragments (− 708--836, − 290—426, − 160--289) in vitro (Fig. 6). We subsequently carried out a dual luciferase reporter assay in tobacco leaves with reporter and effector constructs to examine TaWRKY40-activated *TaGAPC1* promoter activity in vivo. As shown in Fig. 6, the *TaGAPC1* promoter was strongly activated by TaWRKY40. This finding clearly suggested that TaWRKY40 could specifically and directly bind to the W box(C/TTGACC) of the *TaGAPC1*promoter.

### H_2_O_2_ is required for the ABA-induced TaGAPC1 gene expression by PEG8000 treatment

To detect whether the upregulation of *TaGAPC1* under PEG treatment involves the H_2_O_2_ signaling pathway, DMTU was chosen to inhibit of H_2_O_2_ [25]. Wheat plants were pretreated with DMTU for 6 h to stop the production of H_2_O_2_, followed by PEG8000 treatment for 6 h. Figure 7a shows that *TaGAPC1* was induced by PEG (4.61-fold) and H_2_O_2_ (6.93-fold) treatment, consistent with the results in Fig. 1a. Treatment with DMTU reduced the fold increase to 2.11-fold at 6 h after the PEG treatment (Fig. 7a). Treatment with DMTU had no effect on the expression of *TaGAPC1* (Fig. 7a). These results suggested that the upregulation of *TaGAPC1* by PEG8000 treatment possibly involved the H_2_O_2_ signaling pathway.

**Fig. 7:** Effects of inhibitors of ABA and H_2_O_2_ on the *TaGAPC1* transcription under PEG8000 treatment. **a** Effects of pretreatment with inhibitor of H_2_O_2_ on the expression of *TaGAPC1* in the leaves of wheat seedlings exposed to PEG8000. **b** Effects of pretreatment with inhibitor of ABA biosynthesis on the expression of *TaGAPC1* in the leaves of wheat seedlings exposed to PEG8000. **c** Effects of pretreatment with inhibitor of H_2_O_2_ on the expression of *TaGAPC1* in the leaves of wheat seedlings exposed to ABA treatment. Error bars indicate ±SD (*n* = 3, from three technical replicates). Significant differences were assessed with one-sided paired t-tests (*, *P* < 0.05; **, *P* < 0.01). Data in Fig. 7 were derived from experiments that were performed at least three times with similar results, and representative data from one repetition were shown

To explore whether the upregulation of *TaGAPC1* under PEG8000 treatment involves the ABA signaling pathway, tungstate was chosen to inhibit of ABA biosynthesis [26]. Wheat plants were pretreated with tungstate for 6 h followed by PEG8000 treatment. These results clearly showed that *TaGAPC1* was induced at 6 h after the treatment with PEG8000 (4.61-fold) and ABA (6.53-fold) (Fig. 7b), which was in line with the results in Fig. 1a. Pretreatment with the inhibitor of ABA inhibited the upregulation of *TaGAPC1* in the PEG8000-treated wheat seedlings (Fig. 7b). There was no obvious difference in the expression of *TaGAPC1* after treatment with tungstate (Fig. 2a). These results implied that the upregulation of *TaGAPC1* by PEG8000 possibly involved the ABA signaling pathway.

To establish a link between the production of H_2_O_2_ and the expression of *TaGAPC1* in the ABA signaling pathway, wheat plants were pretreated with DMTU, a scavenger for H_2_O_2_, for 6 h, and then exposed to ABA treatment for 6 h. The experimental results showed that pretreatment with DMTU dramatically abolished the expression of *TaGAPC1* induced by ABA (Fig. 2c), suggesting that H_2_O_2_ was required for the ABA-induced upregulation in *TaGAPC1* expression*.*

### The expression of TaGAPC1 is regulated by TaWRKY40 in the ABA signaling pathway

To further investigate the biological activity of TaWRKY40, fused *TaWRKY40*-GFP was transiently expressed in wheat protoplasts. In Fig. 1c, the wheat protoplast expressing 35S:: *TaWRKY40*-GFP showed clear green fluorescence in the nucleus. These results indicated that TaWRKY40 was located in the nucleus. Similar to *TaGAPC1*, the transcription level of *TaWRKY40* was also enhanced in wheat in response to abiotic stresses (10mMH_2_O_2_, 100 μM ABA and 20% PEG8000) (Additional file 2: Figure S2). This finding indicates that *TaGAPC1* and *TaWRKY40* may be involved in a similar signaling pathway. To investigate whether *TaWRKY40* is also involved in the ABA-induced upregulation of *TaGAPC1* expression, wheat protoplasts with transiently overexpressed *TaWRKY40* were used. The relative expression of *TaGAPC1* was significantly higher in the wheat protoplasts of transiently overexpressing *TaWRKY40* than in the control wheat protoplasts. Furthermore, the ABA-induced increase in *TaGAPC1* expression in the control protoplasts was also advanced by the overexpression of the *TaWRKY40* gene under conditions of ABA and mannitol stresses (Fig. 8). These results indicate that these *TaWRKY40* genes are crucial for the ABA-induced upregulation in *TaGAPC1* expression.

**Fig. 8:** *TaWRKY40* gene regulates the expression of *TaGAPC1* in wheat protoplast. The transient overexpression of *TaWRKY40* promoted the ABA-induced expression of *TaGAPC1* in wheat protoplasts. The protoplasts were treated with 100 uM ABA, and the relative expression levels of *TaGAPC1* were analyzed by real-time quantitative RT-PCR. Data in Fig. 8 were derived from experiments that were performed at least three times with similar results, and representative data from one repetition were shown

## Discussion

As a functional conserved enzyme in the cytoplasm, GAPC is involved in the glycolytic pathway of plants, oxidizing glyceraldehyde 3-phosphate to 1,3-diphosphoglycerate. In the past, many studies have focused on the gene expression regulation of plant *GAPDHs*. In Arabidopsis, *GAPC* could be induced by extreme climate and drought stress. In rice, the overexpression of *OsGAPC3* could enhance the salt tolerance [27]. *GAPC* participated in the PA-mediated salt stress responses of Arabidopsis roots [28]. The overexpression of *GAPC* could enhance the drought tolerance of potato (*Solanum tuberosum*) plants [29]. Consistent with previous results in other species [30, 31], the transcription of *TaGAPC1* was significantly induced under PEG, H_2_O_2_, and ABA stress (Fig. 1). Furthermore, the OE Arabidopsis lines had a marked developmental advantage over the WT plants; the survival rate of the OE plants was significantly higher than that of the WT plants after a 25-day drought treatment (Fig. 2). Above all, these results indicate that GAPC is not only the final product of the plant drought resistance pathway, but also an intermediate plant resistance signal due to its specific function and high expression level under abiotic stress conditions.

In general, the association of ROS homeostasis with oxidative stress is well known. Therefore, adjusting ROS homeostasis is necessary to protect plants against the oxidative stress caused by abiotic stresses. Plants have developed mechanisms for eliminating ROS, including the production of enzymatic and nonenzymatic antioxidants. Major enzymatic antioxidants include peroxidase (POD), superoxide dismutase (SOD), catalase (CAT) and ascorbate peroxidase (APX) [23]. It has been reported that GAPC could be a target of H_2_O_2_ [12]. In this study, the decreased levels of H_2_O_2_ and O^2−^ under drought stress in transgenic plants compared with WT plants implied that the ROS scavenging systems of transgenic plants might be more efficient than those of WT plants. Antioxidant enzymes were analyzed, and the activities of SOD and POD were higher in the transgenic lines than in the WT line under drought stress. These results suggested that the overexpression of the *TaGAPC1* gene protected plants against ROS injury by integrating with H_2_O_2_ and enhancing the activation of the antioxidant defence system. When plants suffer from environmental stress, bacterial infection or hormone stimulation, the guard cell signal transduction process is rapidly activated to optimize the ability to absorb CO_2_ and to reduce moisture loss by adjusting stomatal movement [32]. Oxidized GAPC interacts with phospholipase D, increasing the amount of phosphatidic acid, which induces stomatal closure [26]. Consistent with these facts, our preliminary results indicated that the stomatal aperture of the lines overexpressing *TaGAPC1* is smaller than that of wild type under drought condition. (Fig. 3).

Many plant regulators are involved in signal transduction networks during plant growth and development, such as the WRKY transcription factor [33]. *TaWRKY40*, a member of the WRKY family, was identified to interact with the *TaGAPC1* promoter by the yeast one-hybrid assay. The WRKY transcription factor is one of the largest families of transcription factors in plants [34]. When plants are exposed to several stresses, the expression of some WRKY transcription factors is rapidly induced thereby regulating the response to various stresses by participating in several signaling pathways [35, 36]. In Arabidopsis, high temperature treatment induced the expression of *AtWRKY25* and *AtWRKY26*. The overexpression of *AtWRKY25* and *AtWRKY26* enhanced tolerance to heat stress [37]. In wheat, the transcription of *TaWRKY70* was significantly increased under high temperature conditions, as well as under ethylene, salicylic acid and cold (4 °C) stress conditions. In addition, *TaWRKY33* plays a key role in ABA- and drought-responsive signaling networks [38]. Consistent with these reports, the expression of *TaWRKY40* was also increased when wheat was exposed to abiotic stress. The results in Fig. 8 indicate that *TaWRKY40* is crucial for the ABA-induced upregulation in *TaGAPC1* expression. Therefore, when plants are subjected to abiotic stress, *TaWRKY40* bound to the *TaGAPC1* promoter and enhanced promoter activity to increase the *TaGAPC1*gene expression level in the ABA signaling pathway.

## Conclusions

In conclusion, this study revealed that the *TaGAPC1* gene was involved in resistance to abiotic stress and probably the encoded protein acts as a multifunctional protein in addition to its pivotal role in glycolysis. When wheat was subjected to abiotic stress, the inducible transcription factor *TaWRKY40* could bind to the *TaGAPC1* promoter to positively regulate the expression level of *TaGAPC1*gene via the ABA signaling pathway, thereby increasing the stress tolerance of plants under abiotic stress. Future studies investigating the activation mechanism and characterizing *TaGAPC1* in wheat will improve our understanding of this intricate regulatory network and the molecular mechanisms underlying plant abiotic stress, in which GAPCs are involved (Fig. 9).

**Fig. 9:** Working model for *TaGAPC1* in response to drought stress. The expression of *TaWRKY40* is induced by drought stress, then, *TaWRKY40* directly bind to the *TaGAPC1* promoter to positively regulate the expression level of the *TaGAPC1* gene by H_2_O_2_-dependent ABA signaling pathway, thereby increasing the tolerance of plant to drought stress. Among them, (+) represents promotion. Straight lines represent direct effects and dashed lines represent indirect effects

## Methods

### Plant materials and treatments

Wheat (*Triticum aestivum* L.cv. Chinese Spring), tobacco (*Nicotiana tabacum*, cv. NC89) and *Arabidopsis thaliana* (ecotype, Columbia) were used in this study. All seeds were provided by the laboratory of Professor Xi ping Deng of Northwest A&F University. Seeds were grown in a phytotron, which was maintained at a photosynthetic photon flux density (PPFD) of 600 μM m^− 2^·s^− 1^ and 22/23 °C day/night temperature with 16 h light/8 h dark cycles.

The seedling roots were dipped into a solution of 20% PEG8000, 10 mM H_2_O_2_ and 100 μM ABA to examine their response to abiotic stress. All the tissues were sampled at 0, 2, 4, 6, 8, 12 and 24 h. For inhibitor or scavenger treatment, the plants were pretreated with 1 mM tungstate for 6 h and then exposed to 20% PEG8000 for 6 h. The plants were pretreated with 5 mM dimethyl thiourea (DMTU) for 6 h and then exposed to 20% PEG8000 for 6 h. The plants were pretreated with 5 mM dimethyl thiourea (DMTU) for 6 h, and then exposed to 100 μM ABA treatment for 6 h. Treatment with tungstate or DMTU alone was also used as controls in the experiment. Samples from treated or control plants were frozen in liquid nitrogen and stored at − 80 °C until total RNA extraction and qRT-PCR assay. All of the experiments were repeated at least three times.

### Gene expression analysis

Total RNA was isolated from different wheat tissues using the RNAiso plus reagent (TaKaRa, Japan), Realtime PCR and first-strand cDNA synthesis were performed with PrimeScript™ RT-PCR Kit (TaKaRa, Japan), respectively, according to the manufacturer’s instruction. Thereafter, Realtime PCR was performed in optical 96-well plates (BIO plastics, Netherlands) with CFX96 Touch Real-Time PCR Detection System (BIO-RAD, USA) using the SYBR Green method. The expression data was analyzed using the 2-^∆∆Ct^ method. Experiments were repeated at least three times with biologically independent samples. The primers used in this assay were listed in Additional file 3: Table S1.

### Plant transformation

To generate transgenic Arabidopsis plants, the 1014 bp open reading frame of *TaGAPC1* was amplified from wheat cDNA by PCR and cloned into the vector pCAMBIA1302. Arabidopsis plants were transformed using the flower dip method and selected on 1/2 Murashige & Skoog (MS) medium containing 30 μg/mL hygromycin. The hygromycin-resistant T1 seedlings were verified by PCR analysis using specific primers (Additional file 1: Figure S1A) Homozygous T3 seeds were used for experiments.

### Stress tolerance of transgenic Arabidopsis plants

Wild-type and transgenic lines were used for drought tolerance analysis. The seeds were sown on 1/2MS medium containing 30 μg/mL hygromycin for 1 week at 23 °C under a 16 h light/8 h dark cycle. Seedlings similar at growth states were then transplanted into containers filled with soil and watered regularly for 2 weeks. Three-week-old plants were subjected to water withholding for 25 days. One hundred seedlings from each line or control were used to detect survival after 25 days of detained water in one repetition. After 15 days of withholding water, the aboveground parts of seedlings were harvested to measure the contents of H_2_O_2_ and MDA and the activities of POD and SOD and stomatal aperture.

### Analyze of MDA, H_2_O_2_ and antioxidant enzyme activity

Chlorophyll extraction and measurement were performed after extraction in 80% acetone as previously described. Samples were subjected to pigment extraction solution (80% (v/v) acetone, at pH 7.8) for 12 h at 4 °C. The absorbance was read at 663 nm, 647 nm and 537 nm. MDA content was measured by a thiobarbituric acid (TBA) assay as described by Heath & Packer [39]. Samples (0.07 g) were homogenized in a 1 ml 10% (w/v) trichloroaceticacid (TCA) solution on ice. Then the supernatant was collected after centrifuging at 10000хg for 10 min at 4 °C. Next, 400 μL TBA solution (10% (w/v) TCA containing 0.5% TBA (w/v)) was added to a 400 μL supernatant. The mixture was boiled for 30 min in 100 °C water bath. The content of MDA was calculated from the absorbance at 532 nm, 600 nm and 450 nm after centrifugation at 10000хg for 5 min. RWC was measured according to Barr & Weatherley [40]. RWC was calculated from the equation: RWC (%) = [(FW - DW)/(TW - DW)]х100. Fresh weight (FW) of samples was recorded. Afterwards, leaf samples were soaked in distilled water at room temperature for 24 h and were recorded as turgid weight (TW). The samples were then dried (80 °C for 24 h) to obtain the total dry weight (DW).

Nitrotetrazolium blue chloride (NBT) was used to detect O^2−^ [41]. Briefly, Samples were incubated in NBT solution (0.5 mg mL^− 1^ NBT) for 8 h in the dark. Then, chlorophyll was removed using 70% ethanol. NBT polymerization at the site of O^2−^ accumulation produced in a dark blue polymer. H_2_O_2_ content was measured by a KI assay [39]. Samples (0.1 g) were homogenized in a 1 mL 10% (w/v) trichloroaceticacid (TCA) solution on ice. Then the supernatant was collected after centrifuging at 12000хg for 30 min at 4 °C. Next, 400 μL KH_3_PO_4_ solution and 800 μL 1 M KI solution were added to the 400 μL supernatant. The content of H_2_O_2_ was calculated from the absorbance at 390 nm.

Enzyme extraction and measurement were performed as Polle described [42]. For SOD activity, the reaction mixture (100 mM phosphate buffer at pH 7.8, 75 μM nitro blue tetrazolium, 13 mM methionine, 0.1 μM EDTA, 2 μM riboflavin) and enzyme extraction were added to the tube. The tube was shaken with 5000 Lx illuminating for 20 min, and then the absorbance was read at 560 nm. The enzyme activity was expressed as U/g fresh weight. The activity of POD was determined using guaiacol. The enzyme extraction was added to the reaction mixture (0.2 M phosphate buffer at pH 6.0, 50 mM guaiacol, 2% H_2_O_2_). The absorbance was read at 470 nm.

### Stomatal aperture measurement

For the drought-induced stomatal aperture measurements, leaves in the same position on the plant grown for 15 days without water were sampled, and stomata on the leaf were immediately photographed. Stomata of each exfoliated epidermis were photographed using a light EX30 microscope, and the stomatal aperture was measured by Image J software. Stomatal aperture values are presented as means from at least 50 stomata in one repetition.

### Activity analyze of the TaGAPC1 promoter in tobacco

The *TaGAPC1* promoter sequence was inserted into the pC0390-GUS vector and PC0390-RUC to generate recombinant plasmids and then the plasmids were transformed into tobacco leaves by Agrobacterium. The GUS activity was measured with histochemical assays as previously described [43, 44]. A luciferase assay was performed using the Dual-Luciferase Reporter Assay System (Promega) on a GloMax 20/20 Luminometer (Promega) according to the manufacturer’s instructions and our previous descriptions [45, 46].

### Yeast one-hybrid screening

Fragments of the *TaGAPC1* promoter were cloned into plasmid pAbAi to screen the wheat cDNA library. The Yeast One-Hybrid system was performed using the Matchmaker Gold Yeast One-Hybrid Library Screening System from Clontech as recommended by the manufacturer.

### EMSA

An electrophoretic mobility shift assay (EMSA) was performed as previously described with modifications [47, 48]. A total of 40 ng of a 40 bp double stranded probe and 1 μg of purified TaWRKY40 were used in the EMSA reactions. After incubation at room temperature for 30 min, the samples were loaded onto a 6% native polyacrylamide gel and the gel was post-stained with Invitrogen™ SYBR™ Safe DNA Gel Stain and imaged using a BioRad’s gel documentation system to detect DNA.

### Statistical analysis

The results of physiological measurements presented are the means of three independent experiments (biological replicates) analyzed by the SPSS software (IBM analytics, NY, USA). Student’s t-test was performed to determine their significance by LSD at 0.05 probability level.

## Supplementary information

**Additional file 1: Figure S1.** Detection of transgenic plants. (A) Diagram of the 35S:TaGAPC1 constructs. The primers, pr1, pr2 and pr3, used to analyze TaGAPC1 in transgenic Arabidopsis plants were shown. (B, C) PCR analyze of *TaGAPC1* overexpressing transgenic Arabidopsis.

**Additional file 2: Figure S2.** *TaWRKY40* expression in response to abiotic stresses in wheat. Error bars indicate ±SD (*n*=3, from three technical replicates). Significant differences were assessed with one-sided paired t-tests (*, *P* < 0.05; **, *P* < 0.01). Three biological replicates were performed. Data were derived from experiments that were performed at least three times with similar results, and representative data from one repetition were shown.

**Additional file 3: Table S1**. Primer and probe sequences used in this study.

**Additional file 4: Table S2**. Basic local alignment search tool (BLAST) result for potential candidate interacting proteins with *TaGAPC1* promoter in cDNA wheat library.

## Data Availability

The dataset supporting the conclusions of this article is included within the article and its additional files.

## Abbreviations

EMSA: Electrophoretic mobility shift assay
GAPC: Glyceraldehyde-3-phosphate dehydrogenase in cytoplasm
GAPDH: Glyceraldehyde-3-phosphate dehydrogenase
qRT-PCR: Quantitative real time polymerase chain reaction
Y1H: Yeast one-hybrid

## References

[1] Mahajan S, Tuteja N (2005). Cold, salinity and drought stresses: an overview. Arch Biochem Biophys.

[2] Enebe MC, Babalola OO (2018). The influence of plant growth-promoting rhizobacteria in plant tolerance to abiotic stress: a survival strategy. Appl Microbiol Biotechnol.

[3] Nicholls C, Li H, Liu JP (2012). GAPDH: a common enzyme with uncommon functions. Clin Exp Pharmacol Physiol.

[4] Munoz-Bertomeu J, Cascales-Minana B, Mulet J, Baroja-Fernandez E, Pozueta-Romero J, Kuhn J, Segura J, Ros R (2009). Plastidial Glyceraldehyde-3-phosphate dehydrogenase deficiency leads to altered root development and affects the sugar and amino acid balance in Arabidopsis. Plant Physiol.

[5] Jesús M-B, C-Ma B, Asunción I-S, Isabel M, Adriano N-N, Alisdair RF, Juan S, Roc R (2010). The plastidial glyceraldehyde-3-phosphate dehydrogenase is critical for viable pollen development in Arabidopsis. Plant Physiol.

[6] Cerff R, Chambers SE (1979). Subunit structure of higher plant glyceraldehyde-3-phosphate dehydrogenases (EC 1.2.1.12 and EC 1.2.1.13). J Biol Chem.

[7] Martin W, Cerff R (1986). Prokaryotic features of a nucleus-encoded enzyme. FEBS J.

[8] Cerff R, Kloppstech K (1982). Structural diversity and differential light control of mRNAs coding for angiosperm glyceraldehyde-3-phosphate dehydrogenases. Proc Natl Acad Sci U S A.

[9] Muñoz-Bertomeu J, Bermúdez MA, Segura J, Ros R (2011). Arabidopsis plants deficient in plastidial glyceraldehyde-3-phosphate dehydrogenase show alterations in abscisic acid (ABA) signal transduction: interaction between ABA and primary metabolism. J Exp Bot.

[10] Tristan C, Shahani N, Sedlak TW, Sawa A (2011). The diverse functions of GAPDH: views from different subcellular compartments. Cell Signal.

[11] Gani Z, Boradia VM, Ram JR, Suryavanshi PM, Patil P, Kumar S, Singh R, Raje M, Raje CI (2016). Purification and characterization of glyceraldehyde-3-phosphate-dehydrogenase (GAPDH) from pea seeds. Protein Expr Purif.

[12] Hancock JT, Henson D, Nyirenda M (2005). Proteomic identification of glyceraldehyde 3-phosphate dehydrogenase as an inhibitory target of hydrogen peroxide in Arabidopsis. Plant Physiol Biochem.

[13] Muñozbertomeu J, Bermúdez MA, Segura J, Ros R (2011). Arabidopsis plants deficient in plastidial glyceraldehyde-3-phosphate dehydrogenase show alterations in abscisic acid (ABA) signal transduction: interaction between ABA and primary metabolism. J Exp Bot.

[14] Marco V, Mirko Z, Margherita F, Paolo T, Fiorella LS, Alex C (2013). Nuclear accumulation of cytosolic glyceraldehyde-3-phosphate dehydrogenase in cadmium-stressed Arabidopsis roots. Plant Physiol.

[15] Mirko Z, Samuel M, Mariette B, Marchand CH, Margherita F, Nicolas R, Lemaire SD, Paolo T (2013). Mechanisms of nitrosylation and denitrosylation of cytoplasmic glyceraldehyde-3-phosphate dehydrogenase from Arabidopsis thaliana. J Biol Chem.

[16] Peralta DA, Araya A, Gomez-Casati DF, Busi MV (2018). Over-expression of SINAL7 increases biomass and drought tolerance, and also delays senescence in Arabidopsis. J Biotechnol.

[17] Peralta DA, Araya A, Busi MV, Gomez-Casati DF (2016). The E3 ubiquitin-ligase SEVEN IN ABSENTIA like 7 mono-ubiquitinates glyceraldehyde-3-phosphate dehydrogenase 1 isoform in vitro and is required for its nuclear localization in Arabidopsis thaliana. Int J Biochem Cell Biol.

[18] Rius SP, Casati P, Iglesias AA, Gomez-Casati DF (2008). Characterization of Arabidopsis lines deficient in GAPC-1, a cytosolic NAD-dependent glyceraldehyde-3-phosphate dehydrogenase. Plant Physiol.

[19] Zeng L, Deng R, Guo Z, Yang S, Deng X (2016). Genome-wide identification and characterization of Glyceraldehyde-3-phosphate dehydrogenase genes family in wheat ( Triticum aestivum ). BMC Genomics.

[20] Zeng H, Xie Y, Liu G, Lin D, He C, Shi H (2018). Molecular identification of GAPDHs in cassava highlights the antagonism of MeGAPCs and MeATG8s in plant disease resistance against cassava bacterial blight. Plant Mol Biol.

[21] Shaojie H, Yan W, Xiyin Z, Qi J, Jinping Z, Fan B, Yiguo H, Yule L (2015). Cytoplastic Glyceraldehyde-3-phosphate dehydrogenases interact with ATG3 to negatively regulate autophagy and immunity in Nicotiana benthamiana. Plant Cell.

[22] Elizabeth H, Nicholas F, Jun L, Georgia D, Gitta C (2015). Beyond glycolysis: GAPDHs are multi-functional enzymes involved in regulation of ROS, autophagy, and plant immune responses. PLoS Genet.

[23] Gill SS, Tuteja N (2010). Reactive oxygen species and antioxidant machinery in abiotic stress tolerance in crop plants. Plant Physiol Biochem.

[24] Ülker B, Somssich IE (2004). WRKY transcription factors: from DNA binding towards biological function. Curr Opin Plant Biol.

[25] Aying Z, Jun Z, Jianhua Z, Nenghui Y, Hong Z, Mingpu T, Mingyi J (2011). Nitric oxide mediates brassinosteroid-induced ABA biosynthesis involved in oxidative stress tolerance in maize leaves. Plant Cell Physiol.

[26] Guo L, Devaiah SP, Narasimhan R, Pan X, Zhang Y, Zhang W, Wang X (2012). Cytosolic Glyceraldehyde-3-phosphate dehydrogenases interact with phospholipase Dδ to transduce hydrogen peroxide signals in the Arabidopsis response to stress. Plant Cell.

[27] Zhang XH, Rao XL, Shi HT, Li RJ, Lu YT (2011). Overexpression of a cytosolic glyceraldehyde-3-phosphate dehydrogenase gene OsGAPC3 confers salt tolerance in rice. Plant Cell Tissue Organ Culture.

[28] Mcloughlin F, Arisz SA, Dekker HL, Kramer G, Koster CG, De, Haring MA, Munnik T, Testerink C, Identification of novel candidate phosphatidic acid-binding proteins involved in the salt-stress response of *Arabidopsis thaliana* roots. Biochem J 2013, 450(2):573–581.10.1042/BJ2012163923323832

[29] Kappachery S, Baniekal-Hiremath G, Yu JW, Park SW (2015). Effect of over-and under-expression of glyceraldehyde 3-phosphate dehydrogenase on tolerance of plants to water-deficit stress. Plant Cell Tissue Organ Culture.

[30] Yang Y, Kwon HB, Peng HP, Shih MC (1993). Stress responses and metabolic regulation of glyceraldehyde-3-phosphate dehydrogenase genes in Arabidopsis. Plant Physiol.

[31] Russell DA, Sachs MM (1992). Protein synthesis in maize during anaerobic and heat stress. Plant Physiol.

[32] Hetherington AM, F Ian W: The role of stomata in sensing and driving environmental change. Nature 2003, 424(6951):901–908.10.1038/nature0184312931178

[33] Viana VE, Busanello C, Maia LCD, Pegoraro C, De Oliveira AC (2018). Activation of rice WRKY transcription factors: an army of stress fighting soldiers?. Curr Opin Plant Biol.

[34] Oelmüller R. WRKY transcription factors. Trends Plant Sci. 2014.10.1016/j.tplants.2010.02.00620304701

[35] Chen L, Yu S, Li S, Zhang L, Zou C, Yu D (2012). The role of WRKY transcription factors in plant abiotic stresses ☆. Biochim Biophys Acta.

[36] Wang F, Hou X, Wang Z, Wang S, Jiang F, Li Y (2012). A novel cold-inducible gene from Pak-choi (Brassica campestris ssp. chinensis), BcWRKY46, enhances the cold, salt and dehydration stress tolerance in transgenic tobacco. Mol Biol Rep.

[37] Qian-Tang FU: Expression profiles of AtWRKY25,AtWRKY26 and AtWRKY33 under abiotic stresses. Hereditas 2010, 32(8):848–856.10.3724/sp.j.1005.2010.0084820709683

[38] He GH, Xu JY, Wang YX, Liu JM, Li PS, Chen M, Ma YZ, Xu ZS (2016). Drought-responsive WRKY transcription factor genes TaWRKY1 and TaWRKY33 from wheat confer drought and/or heat resistance in Arabidopsis. BMC Plant Biol.

[39] Heath RL, Packer L (1968). Photoperoxidation in isolated chloroplasts : I. kinetics and stoichiometry of fatty acid peroxidation. Arch Biochem Biophys.

[40] Barr HD, Weatherley PE (1962). A reexamination of the relative turgidity technique for estimating water deficit in leaves. Aust J Biol Sci.

[41] Guan Q, Lu X, Zeng H, Zhang Y, Zhu J (2013). Heat stress induction of miR398 triggers a regulatory loop that is critical for thermotolerance in Arabidopsis. Plant J.

[42] Polle A, Otter T, Seifert F (1994). Apoplastic peroxidases and lignification in needles of Norway spruce (Picea abies L.). Plant Physiol.

[43] Jefferson RA (1987). Assaying chimeric genes in plants: the GUS gene fusion system. Plant Mol Biol Report.

[44] Jefferson RA, Kavanagh TA, Bevan MW (1987). GUS fusions: beta-glucuronidase as a sensitive and versatile gene fusion marker in higher plants. EMBO J.

[45] Frey PM, Schärer-Hernández NG, Fütterer J, Potrykus I, Puonti-Kaerlas J (2001). Simultaneous analysis of the bidirectional African cassava mosaic virus promoter activity using two different luciferase genes. Virus Genes.

[46] Díaz-Triviño S, Long Y, Scheres B, Blilou I (2017). Analysis of a plant transcriptional regulatory network using transient expression systems. Methods Mol Biol.

[47] Kim WC, Reca IB, Kim YS, Park S, Thomashow MF, Keegstra K, Han KH (2014). Transcription factors that directly regulate the expression of CSLA9 encoding mannan synthase in Arabidopsis thaliana. Plant Mol Biol.

[48] Ye Y, Wu K, Chen J, Liu Q, Wu Y, Liu B, Fu X (2018). OsSND2, a NAC family transcription factor, is involved in secondary cell wall biosynthesis through regulating MYBs expression in rice. Rice.

